# A Preliminary Study of Alterations in Iron Disposal and Neural Activity in Ischemic Stroke

**DOI:** 10.1155/2022/4552568

**Published:** 2022-08-06

**Authors:** Abolfazl Mahmoudi Aqeel-Abadi, Hamid-Reza Fateh, Saeed Masoudnia, Niloufar Shirzad, Milad Seyfi, Tayyebeh Ebrahimi, Mohammad-Reza Nazem-Zadeh

**Affiliations:** ^1^Medical Physics and Biomedical Engineering Department, Tehran University of Medical Sciences (TUMS), Tehran, Iran; ^2^Department of Physical Medicine and Rehabilitation, Shariati Hospital, Tehran University of Medical Sciences, Tehran, Iran; ^3^Research Center for Molecular and Cellular Imaging, Advanced Medical Technologies and Equipment Institute (AMTEI), Tehran University of Medical Sciences, Tehran, Iran; ^4^Department of Occupational Therapy, School of Rehabilitation, Shahid Beheshti University of Medical Science, Tehran, Iran; ^5^Neuroimaging and Analysis Group (NIAG), Imam Khomeini Hospital Complex, Tehran University of Medical Sciences (TUMS), Tehran, Iran

## Abstract

**Purpose:**

The study aimed to evaluate the postrehabilitation changes in deep gray matter (DGM) nuclei, corticospinal tract (CST), and motor cortex area, involved in motor tasks in patients with ischemic stroke.

**Methods:**

Three patients participated in this study, who had experienced an ischemic stroke on the left side of the brain. They underwent a standard rehabilitation program for four consecutive weeks, including transcranial direct current stimulation (tDCS), neuromuscular electrical stimulation (NMES), and occupational therapy. The patients' motor ability was evaluated by Fugl-Meyer assessment-upper extremity (FMA-UE) and Wolf motor function test (WMFT). Multimodal magnetic resonance imaging (MRI) was acquired from the patients by a 3 Tesla machine before and after the rehabilitation. The magnetic susceptibility changes were examined in DGM nuclei including the bilateral caudate (CA), putamen (PT), globus pallidus (GP), and thalamus (TH) using quantitative susceptibility mapping (QSM). Functional MRI (fMRI) in the motor cortex areas was acquired to evaluate the postrehab functional motor activity. The three-dimensional corticospinal tract (CST) was reconstructed using diffusion-weighted imaging (DWI) and diffusion tensor tractography (DTT), and the fractional anisotropy (FA) was measured along the tract. Ultimately, the relationship between the structural and functional changes was evaluated in CST and motor cortex.

**Results:**

Postrehabilitation FMA-UE and WMFT scores increased for all patients compared to the prerehabilitation. QSM analysis revealed increasing in susceptibility values in GP and CA in all patients at the ipsilesional hemisphere. By fMRI analysis, the ipsilesional hemisphere demonstrated an increase in functional activity in motor areas for all 3 patients. In the ipsilesional hemisphere, the fractional anisotropy (FA) was increased in CST in two patients, while the mean diffusivity (MD) was decreased in CA in a patient, in PT and TH in another patient, and in PT in two patients.

**Conclusion:**

This preliminary study demonstrates that the magnetic susceptibility may decrease at some ipsilesional DGM nuclei after tDCS, NMES, and occupational therapy for patients with ischemic stroke, suggesting a drop in the level of iron deposition, which may be associated with an increase in the level of activity in motor cortex after rehabilitation.

## 1. Introduction

Ischemic stroke accounts for about 80% of all stroke cases, which is one of the leading causes of death and disability worldwide [1, 2]. Patients with ischemic stroke often develop upper limb dysfunction, which results in disability and reduced quality of life [3]. In less than 6 months, about 30-66% of these patients can achieve a relative improvement in the function of their upper limbs, which is often attributed to reduction of cerebral edema and primary neuroplasticity [4]. Recovery after a stroke has two distinguished neurological and functional aspects. Functional recovery is influenced by external environmental factors, continuation of rehabilitation programs, and motivation of the patient, while neurological recovery is determined by the pathogenesis and the blood territory where the stroke onset has occurs [5].

To assess the functional improvement in stroke patients, studies have suggested two impairment indices, i.e., Fugl-Meyer assessment-upper extremity (FMA-UE) and Wolf motor function test (WMFT) [6]. The FMA is a stroke-specific performance-based impairment index, designed to assess motor functioning, balance, sensation, and joint functioning in patients with poststroke hemiplegia. It is applied clinically and in research to determine disease severity, describe motor recovery, and plan and assess treatment [7, 8]. The WMFT quantifies upper extremity movement ability through timed single- or multiple-joint motions and functional tasks [9, 10]. These impairment tests are used to assess patient's ability or to assess recovery [11].

Neuroimaging by magnetic resonance imaging (MRI) is recommended as a complementary method for stroke patients to monitor and evaluate the functional and neurological improvements or declines [12]. MRI can provide morphometric and pathologic information that can assess the functional and neurological improvements. To do this, we need to examine all the areas of the patient's brain that are involved in performing the movements such as motor cortex and deep gray matter (DGM) nuclei that work together to create and control limb movement and are involved in rehabilitation of ischemic stroke patients [13, 14]. It has been shown that the cortex and the corticospinal tract (CST) must also be examined because of the inherent relationships between different areas of the nervous system working together [12], shown in the diagram in Figure 1. In this sequence, the cerebral cortex is the origin of corticospinal fibers and is in charge of voluntary control of fine movements. The basal ganglia play an important role in controlling movement by receiving significant inputs from the cerebral cortex and amplifying and mediating signals to the frontal brain regions. The corticospinal tract arises from three different regions of the cortex including precentral gyrus (referred to as the primary motor cortex or M1), postcentral gyrus (referred to as the primary somatosensory cortex or S1), and the region immediately rostral to the precentral gyrus (supplemental motor area [15] and premotor cortex or PMC) [16, 17] (Figure 1).

Some studies have shown that iron deposition levels in the basal ganglia are significantly altered in patients with vascular disease (dementia and destruction), in particular in ischemic stroke [14, 18–22]. However, it remains unknown whether the metabolism of iron in the basal ganglia would change after a long-term ischemia.

Iron is an important factor for various enzymes involved in neurotransmitter synthesis, oxygen transport, electron transfer, and myelin production. It is stored primarily in the brain tissue as ferritin and hemosiderin to maintain normal brain function [23]. Apart from the essential roles that iron plays in normal physiological functions, its excessive amounts in the brain can lead to the abnormal secretion of toxic free radicals, resulting in oxidative damage [24]. To study the iron deposition, various MRI techniques have been used, most importantly the susceptibility-weighted imaging (SWI) [25] and the quantitative susceptibility mapping (QSM) [26]. They are sensitive to paramagnetic materials, allowing indirect measurement of iron deposition in DGM structures [25, 27, 28] in neurodegenerative diseases [29]. The study of patients with movement disorders and neuronal damages such as stroke by the QSM method with a high accuracy shows the importance of examining the DGM areas as well as the amount of iron deposition in them.

Diffusion-weighted imaging (DWI) is one of the most common noninvasive methods for examining the structure of nerve fibers. DWI is a quantitative MRI technique that examines the movement of water molecules within the microstructures. Valuable diffusion parameters such as fractional anisotropy (FA) and mean diffusivity (MD) can be obtained, which are effective in assessing the integrity of nerve fibers. DWI can be also used to evaluate the integrity of CST fibers that mediated the motor-related activations in the motor cortex areas [13].

Using functional MRI (fMRI), the activity of motor areas can be determined in the brain area undergoing alterations in regional cerebral blood flow [30, 31]. Several studies showed that fMRI can be also used to examine the changes in motor cortex function after ischemic stroke [32–34], as well as to examine the rate of patient's recovery [35, 36].

Few studies have examined stroke only using a couple of these modalities. However, analysis of the entire network involved in a motor task including motor cortical areas, DGM nuclei, and their connections through CST may provide more valuable information about lesion, the rate of improvement, or treatment planning for stroke patients. We addressed previous limitations and examined the rehabilitation process in stroke patients based on both functionally and neurologically evaluations by analysis of clinical and multimodal imaging data and inspecting their relationships.

## 2. Material and Methods

This study was approved by the Research Ethics Committee of Tehran University of Medical Sciences (TUMS), and tacit satisfaction was obtained from all participants. Three patients (2 men and 1 woman, 38-75 Y/O) participated in this study (Table 1). The patients were referred to the rehabilitation center of Shariati Hospital of the TUMS. Ischemic stroke in the patients was confirmed on MRI by a radiologist. All of the patients had the onset in the left brain hemisphere.

### 2.1. Clinical Intervention

First, the patients were evaluated by a therapist for motor injury and upper limb affection using FMA-UE and WMFT tests. Then, they underwent a regular rehabilitation program five days a week for four consecutive weeks. The rehabilitation program included 20 minutes of the brain stimulation with nodal transcranial direct current stimulation (tDCS) with an intensity current of 1.5 mA, neuromuscular electrical stimulation (NMES), and occupational therapy including strengthening, stretching, proprioceptive neuromuscular facilitation (PNF), constraint-induced movement therapy (CIMT), and Brunnstrom movement therapy (BMT). After rehabilitating treatments, FMA-UE and WMFT tests were again completed.

### 2.2. MRI Imaging Protocol

For this study, a 3-Tesla Prisma MRI (Siemens, Germany) located at the National Brain Mapping Laboratory (NBML) and a 64-channel head and neck coil were used. An angled mirror was placed in front of patients so that they could see the display above the patient's head. A head support system and a pad were used to reduce the head movement and motion artifacts.

The patients underwent structural and functional imaging. A 3D T1-weighted image was created using 3D spoiled gradient-recalled (SPGR) sequence with voxel size = 1.1 × 1.1 × 1 mm^3^, TR = 1840.0 ms, TE = 2.13 ms, and total scan time = 4.10 min. For QSM imaging, a 3D gradient-recalled echo (GRE) sequence was used with voxel size = 0.9 × 0.9 × 2.0 mm^3^, TR = 45.0 ms, TE1 = 6.0 ms, number of echoes = 9, distance between echoes = 4 ms, and total scan time = 7 : 24. DWI images were acquired with time of repetition (TR) = 9600 ms, time of echo (TE) = 92.0 ms, voxel size = 2.0 × 2.0 × 2.0 mm^3^, scan time = 5.47 min, number of diffusion directions = 30, bavlue1 = 0, and bvalue2 = 1000/mm^2^. Functional MRI images were obtained using FA = 90 degrees, voxel size = 2.8 × 2.8 × 2.4 mm^3^, TE/TR = 4000/30.0 ms, repeated measurements = 90, and in a total scan time = 6.14 min.

### 2.3. Data Preprocessing

Before diffusion data analysis, a series of preprocessing was performed including extraction and correction of *b* value and *b*-vector and correction of motion artifacts, eddy currents, and distortion. In order to extract the values of activity in the brain areas in the functional data, steps are taken including registration of the functional images on structural image, motion correction, slice timing correction, spatial smoothing, and temporal filtering.

### 2.4. QSM Analysis

The raw phase was unwrapped using Laplacian-based phase unwrapping. The background field was analyzed with a variable-size complex harmonic attenuation kernel (variable-kernel sophisticated harmonic artifact reduction for phase data: V-SHARP) for phase data with a regularization parameter of 0.05 and a maximum radius of 5 mm. Compared to the single-echo technique, we used 9 echoes for a better signal-to-noise ratio. Finally, the inverse bipolar calculation was used using a streaking artifact reduction QSM technique (STAR-QSM) to achieve susceptibility maps. This process is illustrated in Figure 2.

### 2.5. Image Segmentation

We segmented the basal ganglia and thalamus to examine their susceptibility map. First, QSM echo gradient images were registered on T1 using SPM software (http://www.fil.ion.ucl.ac.uk/spm/). T1 and QSM images were used to construct hybrid contrast (HC) images [37], which were then used for segmentation by FSL software (http://www.fmrib.ox.ac.uk/fsl). The extracted masks were used for the segmentation of QSM images. The segmentation process is illustrated in Figure 3, which were finally performed to calculate the magnetic susceptibility indices in the targeted areas. The obtained segmented images are also shown in Figure 4.

### 2.6. Analysis of Motor-Task fMRI and Extraction of Corticospinal Tract

Functional images were obtained from motor tasks for both affected and nonaffected hands. The cerebral cortex associated with movement mainly consists of Brodmann areas of 1 to 6 [38]. The primary motor cortex comprises Brodmann area 4, which is located in and around the precentral gyrus [38, 39]. The primary somatosensory region, on the other hand, includes Brodmann areas 1 to 3 located in and around the postcentral gyrus. The fMRI data were analyzed using FSL software. These areas of the brain were masked, and *t*-statistical values of the activated areas were extracted.

The motor task comprised alternations of a 20-s epoch during which the patients attempted a hand closure (the first epoch began 12 s after initiation of scanning), followed by a 20-s rest epoch. Nine cycles were performed for either hand. The patients were instructed rigorously before starting the task.

DWI of patients was analyzed by ExploreDTI software [40], and the CST was extracted. FA values were calculated along the CST, as well as for DGM regions using AAL (automated anatomical labeling) Atlas [41].

### 2.7. Clinical Assessment

For each patient, FMA and WMFT were taken before and after rehabilitation to assess the upper limb impairment and the upper extremity movement ability, respectively.

## 3. Results

### 3.1. Patient 1

Before rehabilitation, the FMA and WMFT scores were 18 and 12, respectively (Table 1). These scores elevated after rehabilitation to 40 and 15, respectively; which indicates a functional improvement in the patient's movements in the upper limb.

The fMRI activation map of the hand motor task was inspected before and after rehabilitation (Figure 5). The activity level at Brodmann areas of 1, 2, 3, 4, and 6 were extracted. An overall increase in motor activity levels in the ipsilesional (left) hemisphere was seen, with no obvious change on the contralesional (right) hemisphere (Figure 6(a)).

In the DWI study, FA and MD indices in CST were illustrated in Figure 7. As shown, a noticeable increase in bilateral CST was observed in both volume and length of the CST (Figure 8), with a dominant decrease at ipsilesional hemisphere (left). The MD values extracted from DGM nuclei areas showed a bilateral decrease in CA (Figure 9(a)). The FA values in ipsilesional CST was slightly increased after rehabilitation (Figure 10).

QSM analysis demonstrated a decrease in susceptibility values in nuclei of PT, GP, CA, and TH, indicating a decrease in iron deposition level in DMG nuclei (Figure 11(a)).

### 3.2. Patient 2

The FMA and WMFT scores were increased from 4 and 5 (before rehabilitation) to 8 and 10 (after rehabilitation), respectively (Table 1), indicating a functional improvement in patient's movement. Based on fMRI analysis, a significant increase in motor activity was observed in all ipsilesional motor cortex areas after rehabilitation (functional activity in Brodmann areas is shown in Figure 6(b)). Although a moderate increase in activity was observed in most areas on the contralesional hemisphere, activities in some areas including BA3bR, BA3aR, and BA2R were decreased after rehabilitation.

By the DWI analysis, MD values decreased in right TH and left PT (Figure 9(b)). We also observed a decrease in FA values of the CST, bilaterally (Figure 10).

Figure 11(b) shows the QSM analysis results for patient 2, where a decrease in susceptibility values of all ipsilesional nuclei was seen, indicating a global decrease in iron deposition level in the ipsilesional hemisphere. In the contralesional hemisphere, a decrease was observed in PT and TH.

### 3.3. Patient 3

Before rehabilitation, FMA and WMFT values were 8 and 2, respectively. After rehabilitation, these scores elevated to 14 and 6, respectively (Table 1), confirming an improvement in patient's movements. Based on fMRI analysis, the activations in almost all ipsilesional motor areas increased (Figure 6(c)). However, no consistent change was observed in the contralesional hemisphere.

In the DWI study, MD value showed a decrease in bilateral TH and PT and in contralesional GP (Figure 9(c)). The FA value in the CST increased bilaterally (Figure 10). The QSM analysis demonstrated a decrease in susceptibility values in bilateral GP and CA nuclei and in contralesional putamen (Figure 11(c)).

The analysis of patients' functional and neurological recovery assessment in this study can be summarized as follows. Functional recovery was assessed by the FMA and WMFT tests, which showed an elevation in all patients and confirmed the efficacy of rehabilitation process. The fMRI analysis also showed increased activations at all ipsilesional motor areas after rehabilitation (Table 2). However, no consistent change was generally observed in the contralesional hemisphere. In two patients, we observed an increase in the FA value of the ipsilesional CST (Table 2). The pre- versus postrehabilitation data analysis of QSM images in DGM nuclei showed a decrease in the average susceptibility values at the ipsilesional hemisphere (Table 2). We observed a reduction in the average MD values for two patients in DGM nuclei (Table 2).

## 4. Discussion

The aim of this study was to evaluate the alterations of iron deposition (magnetic susceptibility) in the basal ganglia and thalamus in ischemic stroke patients and to assess the importance of multimodal imaging and the correlation between different MRI image modalities in this domain. We used neuroimaging data including QSM, DWI, and fMRI, as well as FMA and WMFT clinical tests to evaluate the neural basis of the recovery after rehabilitation in ischemic stroke patients. All three patients were right-handed and had a lesion on the left side of their brain that caused a movement defect in the right limb.

We observed a decrease in the magnetic susceptibility in DGM regions, an increase in FA values within corticospinal tract, and an increase in fMRI activations in motor cortex areas, as well as an improvement in FMA and WMFT clinical tests. More specifically, by inspection of the QSM images of these patients after rehabilitation, two of the patients underwent a decrease in the magnetic susceptibility in all ipsilesional basal ganglia, but for a patient, we only observed a decrease in GP and CA, bilaterally. In general, in all three patients, the neuroimaging analysis implied a decrease in iron deposition level in GP and CA.

The CST is the main neural pathway that provides the function of voluntary movement. This tract attaches the cortex to the spinal cord and activates limb movement. CST preservation and recovery are essential for improvement of motor dysfunction following a brain injury [42]. Studies have shown that the degree of movement disturbance during ischemic stroke depends on the amount of CST affection within the ischemic onset [43]. Patients with a higher recovery after an ischemic stroke showed a greater CST integration compared to those with an insignificant recovery after rehabilitation [44]. In cases experiencing reduced FA values, the nerve fibers are mostly demyelinated and damaged. In contrast, a reduction in MD value implies that the diffusivity of the water molecules is restricted, and the nerve cells are in a better integrity [45, 46]; thus, the DWI can be used to study the integrity of nerve fibers in ischemia and evaluate the level of brain damage [45–49]. Previous studies have shown that DWI and more specifically the FA index can be used to assess the extent of damage to the corticospinal tract [31, 33]. They suggested that the severity of the damage to the motor areas may be correlated to the amount of decrease in FA values [50]. Our results were in line with previous findings, i.e., where the increased FA values in the ipsilesional corticospinal tract in two of the patients were correlated with the increase of fMRI activation.

There is growing evidence from human brain imaging studies that a partial recovery in the movement of an affected limb after a stroke is associated with an altered activity in motor cortical regions [51, 52]. fMRI can look at the connection between the cerebral cortex and subcortical components. Findings also show that improvement of motor performance would be accompanied with reinforcing integrity in CST, depending on the ability and the participation level of the motor cortex in functional motor tasks [53]. In this study, we also observed that for all three patients, the functional activity in the ipsilesional cortex increased after rehabilitation.

Our result was consistent with reported findings in previous studies [14, 18, 29, 54–57], where an increase in iron deposition level in basal ganglia and thalamus were confirmed poststroke. However, only Gattringer et al. [58] did not observe a relationship between the damage severity and the increased iron deposition in DGM regions.

We observed partial improvements in the contralesional brain hemisphere, maybe due to an active reorganization [50, 59, 60]. There are also studies showing that motor performance is related to the amount of iron in the basal ganglia [56]. In our study, in all three patients, iron deposition level was decreased after rehabilitation accompanied with increasing the motor activation in fMRI, with a negative correlation.

Similar to previous studies, our results of FMA and WMFT tests confirmed the improvement of all patients' motor ability and recovery after the rehabilitation process [6, 11]. The fMRI findings were also consistent with the improvements, where we observed an increase in motor activation in all ipsilesional motor areas (except in BA3aL region of a patient). We did not observe a consistent finding at the contralesional hemisphere after rehabilitation.

Recent studies have also pointed to the association between increasing the iron deposition in DGM nuclei and increasing in MD values [61]. A decrease in MD value was observed in the ipsilesional CA in a patient and in PT in another patient.

Previous studies have shown that the ischemic stroke patients often undergo only a couple of these modalities, including studies of the basal ganglia, motor cortex, or CST [11, 14, 30, 31, 33–36, 38–40, 43–45, 47], or the FMA and WMFT clinical tests [8–11]. Only a recent study [49] has evidenced an association between increased iron deposition in DGM nuclei and poor motor performance. Except the recent study, all previous studies only evaluated a few brain areas using a limited number of imaging modalities.

The most important limitation of this study was the number of patients participating in imaging and rehabilitation program due to the pandemic COVID-19. Further studies are required to establish the finding of this work in a statistical cohort analysis.

## 5. Conclusion

Despite recruiting a quite small sample size, this preliminary work has demonstrated that multimodal imaging and clinical tests are associated with one another; each has specific viewpoint to brain changes after stroke and rehabilitation. In order to assess patient's recovery, all the evidence and findings should be considered. We emphasize that the results of DWI and fMRI can monitor and confirm the rate of improvement in stroke patients. Hence, it is not sufficient to rely on just one modality. Magnetic susceptibility mapping and diffusion MRI can be also used to quantify the patient's physiological recovery after rehabilitation.

## Figures and Tables

**Figure 1:** The basal ganglia and thalamus and their relationship to the motor cortex.

**Figure 2:** Illustration of STAR-QSM technique. The raw phase was unwrapped using Laplacian-based phase unwrapping. The background field was analyzed with a complex harmonic variable size kernel of V-SHARP attenuation for phase data with a regularization parameter of 0.05 and a maximum radius of 5 mm. Note: STAR-QSM: streaking artifact reduction quantitative susceptibility mapping; V-SHARP: variable-kernel sophisticated harmonic artifact reduction for phase.

**Figure 3:** Image segmentation pipeline for producing the hybrid contrast images. First, the registration transfer matrix is computed based on magnitude GRE images, and the QSM images are reconstructed based on the phase images. HC images are then produced using T1 and QSM images. At the last step, HC images are segmented using FSL_FIRST, and the masks of DGM regions are finally achieved. Note: DGM: deep gray matter; GRE: gradient-recalled echo; HC: hybrid contrast; MNI: Montreal Neurological Institute; QSM: quantitative susceptibility mapping.

**Figure 4:** Illustration of the segmented basal ganglia on HC images (axial (a) and coronal (c) views), on QSM images (axial (b) and coronal (d) views), and their 3D rendering (e to h). Note: HC: hybrid contrast; QSM: quantitative susceptibility mapping. Color assignment to brain structures: yellow: caudate nucleus; green: putamen; pink: globus pallidus; cyan: thalamus; red: hippocampus; blue: amygdala; brown: nucleus accumbens.

**Figure 5:** fMRI activation map for patient 1 undergoing the motor hand task, for left hand (unaffected hand) before rehabilitation (a); right hand (affected one) before rehabilitation (b); left hand after rehabilitation (c); and right hand after rehabilitation (d).

**Figure 6:** The level of fMRI activity extracted from Brodmann areas 1, 2, 3, 4, and 6 in patients 1, 2, and 3. After rehabilitation, an increase in activity is seen in all the motor cortex areas in patient 1 (a), in all ipsilesional (left) motor cortex areas in patient 2 (b), and in all ipsilesional (left) motor cortex areas, except for BA3aL in patient 3 (c).

**Figure 7:** T1-w images, FA maps, and MD maps of patient 1 before (pre) and after (post) rehabilitation. Note: FA: fractional anisotropy; MD: mean diffusivity.

**Figure 8:** Extracted CST in axial (a) and coronal views (b) before (pre) and after (post) rehabilitation for patient 1. Note: CST: corticospinal tract.

**Figure 9:** Mean diffusivity (MD) values in deep gray matter nuclei in patients 1, 2, and 3. After rehabilitation, no visible change is observed for patient 1 (a), while a slight decrease is observed in ipsilesional (left) thalamus in patient 2 (b) and in the thalamus and putamen for patient 3 (c).

**Figure 10:** Fractional anisotropy (FA) values in left and right corticospinal tract (CST) in patients (pt1, pt2, and pt3). After rehabilitation, a slight increase in ipsilesional (left) CST is observed in patients 1 and 3.

**Figure 11:** The susceptibility values extracted from DGM nuclei areas in patients 1, 2, and 3. After rehabilitation, a slight decrease is observed in ipsilesional (left) hemisphere for the patients 1 and 2 (a) and (b), and in ipsilesional CA and GP for the patient 3 (c). Note: DGM: deep gray matter; PT: putamen; CA: caudate; TH: thalamus; GP: globus pallidus.

**Table 1:** The patient characteristics and clinical data.

Patient	Sex	Age (Y)	Lesion side (brain)	Handedness	Poststroke (month)	Fugl-Meyer assessment (FMA)		Wolf motor function test (WMFT)	
						Pre	Post	Pre	Post
1	M	38	L	R	2	18	40	12	15
2	M	75	L	R	2	4	8	5	10
3	F	68	L	R	6	8	14	2	6

M = male; F = female; L = left; R = right; pre = prerehabilitation; post = postrehabilitation.

**Table 2:** The changes detected by different imaging modalities after rehabilitation in ipsilesional hemisphere.

Patient number	Modality	CA	PT	GP	TH	Motor cortex	CST
Patient 1	QSM	-0.008	-0.002	-0.014	-0.002		
	MD	-4.07	0.30	0.71	0		
	fMRI					2.055	
	FA						0.007

Patient 2	QSM	-0.010	-0.013	-0.020	-0.004		
	MD	0.03	-1.04	1.02	11.8		
	fMRI					2.43	
	FA						-0.015

Patient 3	QSM	-0.052	0.021	-0.050	0.005		
	MD	12.2	-4.02	8.86	-34		
	fMRI					2.05	
	FA						0.028

Note: CA: caudate; PT: putamen; GP: globus pallidus; TH: thalamus; CST: corticospinal tract; FA: fractional anisotropy; MD: mean diffusivity; QSM: quantitative susceptibility mapping.

## Data Availability

The stroke data used to support the findings of this study are available from the corresponding author upon request.

## Abbreviations

BMT: Brunnstrom movement therapy
CA: Caudate
CIMT: Constraint-induced movement therapy
CST: Corticospinal tract
DGM: Deep gray matter
DTT: Diffusion tensor tractography
DWI: Diffusion-weighted imaging
GRE: Gradient-recalled echo
FA: Fractional anisotropy
FMA-UE: Fugl-Meyer assessment-upper extremity
HC: Hybrid contrast
GP: Globus pallidus
M1: Primary motor cortex
MD: Mean diffusivity
MNI: Montreal neurological institute
MRI: Magnetic resonance imaging
NMES: Neuromuscular electrical stimulation
PMC: Premotor cortex
PNF: Proprioceptive neuromuscular facilitation
PT: Putamen
QSM: Quantitative susceptibility mapping
S1: Primary somatosensory cortex
SPGR: Spoiled gradient-recalled
STAR-QSM: Streaking artifact reduction quantitative susceptibility mapping
SWI: Susceptibility-weighted imaging
tDCS: Transcranial direct current stimulation
TH: Thalamus
TE: Time of echo
TR: Time of repetition
V-SHARP: Variable-kernel sophisticated harmonic artifact reduction
WMFT: Wolf motor function test.
